# Comparison of Dopamine and Norepinephrine Use for the Treatment of Hypotension in Out-Of-Hospital Cardiac Arrest Patients with Return of Spontaneous Circulation

**DOI:** 10.1155/2020/7951025

**Published:** 2020-08-18

**Authors:** Chao-Jui Li, Kuan-Han Wu, Chien-Chih Chen, Yat-Yin Law, Po-Chun Chuang, Yi-Chuan Chen

**Affiliations:** ^1^Department of Emergency Medicine, Kaohsiung Chang Gung Memorial Hospital, Chang Gung University College of Medicine, Kaohsiung, Taiwan; ^2^Institute of Medicine, Chung Shan Medical University, Taichung, Taiwan; ^3^Department of Orthopedics, Chung Shan Medical University Hospital, Taichung, Taiwan; ^4^Department of Emergency Medicine, Chang Gung Memorial Hospital, No. 6 W. Sec., Jiapu Rd., Puzih, Chiayi County 613, Taiwan; ^5^Department of Nursing, Chang Gung University of Science and Technology, Chiayi Campus, Chiayi, Taiwan

## Abstract

In patients experiencing out-of-hospital cardiac arrest (OHCA), hypotension is common after return of spontaneous circulation (ROSC). Both dopamine and norepinephrine are recommended as inotropic therapeutic agents. This study aimed to determine the impact of the use of these two medications on hypotension. This is a multicenter retrospective cohort study. OHCA patients with ROSC were divided into three groups according to the post resuscitation inotropic agent used for treatment in the emergency department, namely, dopamine, norepinephrine, and dopamine and norepinephrine combined therapy. Thirty-day survival and favorable neurologic performance were analyzed among the three study groups. The 30-day survival and favorable neurologic performance rates in the three study groups were 12.5%, 13.0%, and 6.8% as well as 4.9%, 4.3%, and 1.2%, respectively. On controlling the potential confounding factors by logistic regression, there was no difference between dopamine and norepinephrine treatment in survival and neurologic performance (adjusted odds ratio (aOR): 1.0, 95% confidence interval (CI) 0.48–2.06; aOR: 0.8, 95% CI: 0.28–2.53). The dopamine and norepinephrine combined treatment group had worse outcome (aOR: 0.6, 95% CI: 0.35–1.18; aOR: 0.2, 95% CI: 0.05–0.89). In conclusion, there was no significant difference in post-ROSC hypotension treatment between dopamine and norepinephrine in 30-day survival and favorable neurologic performance rates.

## 1. Introduction

In patients developing out-of-hospital cardiac arrest (OHCA), hypotension often occurs within minutes to hours of return of spontaneous circulation (ROSC) [1, 2]. Post-ROSC hypotension is a predictor of in-hospital death and is associated with diminished functional status among survivors [3, 4]. Therefore, post-ROSC hypotension should be treated aggressively. Dopamine and norepinephrine are both commonly used inotropic therapeutic agents for hypotension [5]. Norepinephrine is a naturally occurring potent vasoconstrictor and an inotropic agent. Dopamine is a catecholamine-like agent and a chemical precursor of norepinephrine that has both *α*-receptor- and *β*-receptor-stimulating actions. Currently, Backer et al. reported that the use of dopamine was associated with a greater number of adverse events for shock patients [5]. In patients with septic shock, norepinephrine is preferred to dopamine. This is because dopamine is associated with greater mortality and has a higher incidence of arrhythmic events than that of norepinephrine [6]. However, there is no evidence demonstrating the superiority of any one vasopressor in the postcardiac arrest patient. In this study, we aimed to determine the impact of the use of dopamine and norepinephrine on hypotension in ROSC patients.

## 2. Materials and Methods

This multicenter retrospective cohort study was approved by the Institutional Review Board of the Chang Gung Medical Foundation (201600794B0). All patients' records and information were anonymized and deidentified before analysis.

This study was conducted in five emergency departments (EDs) within the same healthcare system in Taiwan, between January 2010 and December 2014. Two EDs were located in a tertiary referral medical center, whereas the other three were situated in secondary regional hospitals. All adult patients (older than 18 years old) who presented to the EDs with nontraumatic cardiac arrest and developed sustained ROSC (when chest compressions are not required for 20 consecutive minutes and signs of circulation persist) with inotropic agent therapy (dopamine or norepinephrine) were included in this study [7, 8]. Patients with a do-not-resuscitation order were excluded.

Demographic data and baseline medical conditions related to Charlson comorbidity index [9], including a history of myocardial infarction, heart failure, cerebrovascular accident, chronic obstructive pulmonary disease, renal and liver disease, and malignancy as well as ED resuscitation records, were extracted from the ED administrative database of participating hospitals [10].

In the five EDs, OHCA patients developing post-ROSC hypotension were treated according to the standard advanced cardiovascular life support (ACLS) protocol. Patients were divided into three groups according to the postresuscitation inotropic agent used in EDs, namely, dopamine, norepinephrine, and dopamine and norepinephrine combined therapy. The primary outcome was 30-day survival. The secondary outcome was favorable neurologic performance, which was according to the Cerebral Performance Category (CPC), with scores 1 and 2 [7]. Two other resuscitation medication doses including epinephrine and sodium bicarbonate were also counted. The dose of epinephrine was 1 mg per vial and that of sodium bicarbonate was 16.7 meq per vial. The relationships between the three study groups and primary and secondary outcomes and the two resuscitation medications were analyzed.

For continuous variables, the data were summarized as means and standard deviations (SD) or medians with interquartile ranges (IQRs) if the data were not normally distributed. The categorical demographic factors were presented as numbers and percentages. Analysis of variance, nonparametric Kruskal–Wallis, and chi-squared tests were used for analyses. To control the potential confounding factors, binomial and multinomial logistic regression analyses were conducted to analyze the relationship between inotropic agent therapy and outcome and the association between inotropic agent therapy and epinephrine and sodium bicarbonate. The effects were estimated in terms of adjusted odds ratios (aORs) and the corresponding 95% confidence intervals (CIs). Significance testing was two-sided, and *p* < 0.05 was considered to indicate statistical significance. SPSS version 12.0 (SPSS, Chicago, IL) was used for all statistical analyses.

## 3. Results

In total, 7410 nontraumatic OHCA patients visited the five EDs during the study period. Among them, 1434 (19.4%) developed ROSC, and 1011 (13.6%) developed post-ROSC hypotension. Among the posthypotension patients, 669 (66.2%) survived to intensive care unit (ICU) admission, and 225 had 30-day survival. Patients who developed ROSC were divided into three treatment groups (Figure 1). There were 670 with dopamine, 92 with norepinephrine, and 249 with dopamine and norepinephrine combined therapy.  Table 1 shows patients' demographics, comobility, Charlson Comorbidity Index, status upon arrival, and treatment type in the EDs in the three study groups. Figures 2 and 3 show the survival curve and the rates of 30-day survival and favorable neurologic performance. While patients who needed both dopamine and norepinephrine combined therapy after resuscitation had worse survival rate and neurologic outcome, the outcomes in the dopamine and norepinephrine groups were similar.

To control the potential confounding factors, binomial logistic regression analyses were conducted.  Table 2 shows the outcome of regression. With increasing age, patients tended to have a lower survival rate and poorer neurologic outcome. Patients presenting to EDs with shockable rhythms had higher a 30-day survival rate but no more favorable neurologic result. Increasing use of epinephrine and sodium bicarbonate was associated with lower 30-day survival but not related to good neurologic performance. Finally, during the postresuscitation period, compared with patients who received dopamine treatment alone, patients who needed both dopamine and norepinephrine combined therapy had a poor neurologic outcome. There was no significant difference between patients who used dopamine and norepinephrine.

Table 3 shows the relationship between resuscitation medications (epinephrine and sodium bicarbonate) and postresuscitation inotropic agent therapy. Patients receiving more sodium bicarbonate therapy had a higher chance of requiring dopamine and norepinephrine combined therapy during the postresuscitation period.

## 4. Discussion

ROSC after OHCA is characterized by myocardial stunning and a robust systemic proinflammatory response [11]. Trzeciak et al. reported that post-ROSC hypotension is a predictor of in-hospital death and is associated with diminished functional status among survivors [3]. This finding is in line with that of our research. Clinically, increased use of inotropic agents during the postresuscitation period indicated that these patients had a more unstable haemodynamic presentation. In our study, patients who needed both dopamine and norepinephrine after ROSC had lower 30-day survival and favorable neurologic performance rates than those who needed only one inotropic agent. We believe that it might be related because these patients were sicker than those in the other groups. On the other hand, the overall survival rate was obviously lower in our study, and this might partially be due to the type of study population. Stephen et al. reported the data of patients admitted to the ICU. In our study, only 66.2% patients had survival to ICU admission. This might have influenced the outcome.

Recently, some studies suggested norepinephrine is superior to dopamine for the treatment of shock. Backer et al. reported an increased 28-day mortality among patients with cardiogenic shock when treated with dopamine as compared with that in treatment with norepinephrine [5]. A meta-analysis reported that dopamine, compared with norepinephrine, was associated with a higher incidence of arrhythmias and with an increased risk of death in patients with septic shock [6]. Rui et al. reported that norepinephrine was associated with a lower 28-day mortality, lower risk of arrhythmic events, and gastrointestinal reaction [12]. There was no suggestion about post-ROSC hypotension. According to our study, when comparing the 30-day survival and favorable neurologic outcome between the dopamine and norepinephrine groups, there was no significant difference. However, in our study, fewer patients were treated with norepinephrine than those treated with dopamine. The reason for why there were more patients given dopamine as compared with receiving norepinephrine is that, in general, dopamine is the first line vasopressor that would be used amongst practitioners of the 5 emergency departments involved in our study. This might have influenced the analysis of the outcome.

Post-ROSC therapy is a crucial link in the “Chain of Survival” paradigm for treating cardiac arrest [13]. However, some types of resuscitation treatments might also influence the post-ROSC hemodynamic performance. Prolonged ventricular fibrillation is related to postresuscitation hypotension [14]. Severe metabolic acidosis is associated with refractory shock [15]. In our study, we counted the dose of epinephrine and sodium bicarbonate. The epinephrine dose is related to the resuscitation duration, and sodium bicarbonate is associated with the degree of acidosis. Owing to the retrospective nature of the study, which is a potential limitation, the data of some parameters such as cardiopulmonary resuscitation duration and blood gas analysis were not available in the medical records, but information on the two medications might provide us further important information. Patients who received more sodium bicarbonate had higher chance of needing combined inotropic agent use. These findings were also compatible with those of the previous research in this area.

There are some limitations of this study. The retrospective nature of the study made it difficult to assemble the data; hence, there was no stratified analysis according to the etiology. There was no prehospital information and long-term follow-up after discharge. In the study hospitals, prehospital information was not included as part of hospital electronic medical records; therefore, the analysis did not consider this. However, some patients were not brought by emergency medical technicians, but by their family; they might not have received basic life support during transportation. Treating postcardiac arrest hypotension should include fluid resuscitation, but we did not have data about fluid treatment. We did not know the total inotropic dose which patients received and intravenous (IV) route either. Unlike epinephrine which is administered often as an IV shot during resuscitation, dopamine and norepinephrine administration was a continuous IV drip, making it difficult to calculate the dose. We had no laboratory data and vital signs before and after each treatment, and the number of patients who received norepinephrine therapy was much fewer than that in the other study groups which might have influenced the data analysis. Finally, although it was a multicenter study, the five study EDs belonged to the same healthcare system, potentially limiting the implications of the results.

## 5. Conclusions

In conclusion, our study did not show any significant difference in post-ROSC hypotension treatment between dopamine and norepinephrine in 30-day survival rate and favorable neurologic performance. Patients needing combined inotropic agents had poor prognosis. Increasing use of bicarbonate during resuscitation was associated with post-ROSC hypotension needing combined inotropic agent therapy.

## Figures and Tables

**Figure 1:** Flowchart of the patient selection process. The patients were included in the study based on the criteria shown above and were divided into three treatment groups.

**Figure 2:** Survival curves of the three treatment groups. Compared with the dopamine treatment group (blue line), the *p* values were 0.128 (norepinephrine) (green line) and 0.002 (dopamine + norepinephrine) (gray line).

**Figure 3:** Thirty-day survival and favorable neurologic performance rates in the three study groups. Thirty-day survival rates: 12.1%, 13.0%, and 6.0% (*p*=0.022); favorable neurologic performances: 4.9%, 4.3%, and 1.2% (*p*=0.036).

**Table 1:** Characteristics of patients treated with different inotropic agents after return of spontaneous circulation.

	Dopamine (*n* = 670)	Norepinephrine (*n* = 92)	Dopamine + Norepinephrine (*n* = 249)	*p*-value
Age	68.7 ± 15.87	66.4 ± 18.02	68.1 ± 16.26	0.438
Male	367 (54.8%)	52 (56.5%)	138 (55.4%)	0.989

Comobility				
Heart failure	92 (13.7%)	10 (10.9%)	26 (10.4%)	0.355
CVA	136 (20.3%)	25 (27.2%)	53 (21.3%)	0.318
COPD	165 (24.6%)	16 (17.4%)	47 (18.9%)	0.083
DM	194 (29.0%)	32 (34.8%)	84 (33.7%)	0.252
Renal disease	131 (19.6%)	11 (12.0%)	33 (13.3%)	0.029
Liver cirrhosis	85 (12.7%)	11 (12.0%)	30 (12.0%)	0.955
Malignancy	89 (13.3%)	13 (14.1%)	40 (16.1%)	0.559
CCI	3 ± 1.5	2 ± 2.0	3 ± 1.5	0.574

*Status upon arrival*				
EMT transfer	482 (71.9%)	73 (79.3%)	178 (71.5%)	0.302
Shockable rhythm	71 (10.6%)	14 (15.2%)	21 (8.4%)	0.190

Treatment in ED				
Epinephrine (mg)	5 ± 2.5	5 ± 2.0	7 ± 3.5	<0.001
Sodium bicarbonate (vial)	4 ± 4.0	4 ± 4.5	8 ± 5.0	<0.001
PCI	28 (4.2%)	4 (4.3%)	5 (2.0%)	0.278
ECMO	7 (1.0%)	2 (2.2%)	1 (0.4%)	0.330
ICU admission	475 (70.9%)	66 (71.7%)	146 (58.6%)	0.001

CVA: cerebrovascular accident; COPD: chronic obstruction pulmonary disease; DM: diabetes mellitus; EMT: emergency medical technician; shockable rhythm: ventricular fibrillation and pulseless ventricular tachycardia; ED: emergency department; PCI: percutaneous coronary intervention; ECMO: extracorporeal membrane oxygenation; ICU: intensive care unit.

**Table 2:** Association of postresuscitation inotropic agent therapy and 30-day survival and favorable neurologic performance.

	30-day survival		Favorable neurologic performance	
	aOR	95% C.I.	aOR	95% C.I.
Age	0.96	0.942∼0.972	0.95	0.929∼0.974
Male	1.0	0.65∼1.67	1.8	0.84∼3.90
Charlson comorbidity index	1.0	0.91∼1.12	1.0	0.87∼1.20
Shockable rhythm	2.1	1.12∼4.11	1.6	0.56∼4.35
Epinephrine	0.9	0.89∼0.99	1.0	0.88∼1.04
Sodium bicarbonate	0.95	0.912∼0.996	1.0	0.94∼1.06

*Postresuscitation inotropic therapy*				
Dopamine	1			1
Norepinephrine	1.0	0.48∼2.06	0.8	0.28∼2.53
Dopamine + norepinephrine	0.6	0.30∼1.10	0.2	0.04∼0.78

Shockable rhythm: ventricular fibrillation and pulseless ventricular tachycardia; aOR: adjusted odds ratio; CI: confidence interval.

**Table 3:** Association between postresuscitation inotropic agent therapy and resuscitation medication.

	Dopamine		Norepinephrine		Dopamine + norepinephrine	
	aOR	95% C.I.	aOR	95% C.I.	aOR	95% C.I.
Epinephrine	1	—	1.0	0.90∼1.02	1.0	1.00∼1.06
Sodium bicarbonate	1	—	1.0	0.95∼1.04	1.1	1.05∼1.11

Adjusted for age, sex, Charlson Comorbidity Index, and cardiac rhythm in multinomial logistic regression. aOR: adjusted odds ratio; CI: confidence interval.

## Data Availability

The data used to support the findings of this study have not been made available, because, according to the policy of the Institutional Review Board of the Chang Gung Medical Foundation, the patients' data should not be made publicly available.
